# Screening Potential Diagnostic Biomarkers for Age-Related Sarcopenia in the Elderly Population by WGCNA and LASSO

**DOI:** 10.1155/2022/7483911

**Published:** 2022-09-13

**Authors:** Shangjin Lin, Ming Ling, Cong Chen, Xiaoxi Cai, Fengjian Yang, Yongqian Fan

**Affiliations:** ^1^Department of Orthopedics, Huadong Hospital Affiliated to Fudan University, Shanghai 200040, China; ^2^Shanghai Key Laboratory of Clinical Geriatric Medicine, Shanghai 200040, China

## Abstract

**Background:**

Sarcopenia is a common chronic disease characterized by age-related decline in skeletal muscle mass and function, and the lack of diagnostic biomarkers makes community-based screening problematic.

**Methods:**

Three gene expression profiles related with sarcopenia were downloaded and merged by searching the Gene Expression Omnibus (GEO) database. Differentially expressed genes (DEGs) and eigengenes of a module in the merged dataset were identified by differential expression analysis and weighted gene coexpression network analysis (WGCNA), and common genes (CGs) were defined as the intersection of DEGs and eigengenes of a module. CGs were subjected to gene ontology (GO) and Kyoto Encyclopedia of Genes and Genomes (KEGG) enrichment analysis. Subsequently, the least absolute shrinkage and selection operator (LASSO) analysis was performed to screen the CGs for identifying the diagnostic biomarkers of sarcopenia. Based on the diagnostic biomarkers, we established a novel nomogram model of sarcopenia. At last, we validated the diagnostic biomarkers and evaluated the diagnostic performance of the nomogram model by the area under curve (AUC) value.

**Results:**

We screened out 107 DEGs and 788 eigengenes in the turquoise module, and 72 genes were selected as CGs of sarcopenia by intersection. GO analysis showed that CGs were mainly involved in metal ion detoxification and mitochondrial structure, and KEGG analysis revealed that CGs were mainly enriched in the mineral absorption, glucagon signaling pathway, FoxO signaling pathway, insulin signaling pathway, AMPK signaling pathway, and estrogen signaling pathway. Then, six diagnostic biomarkers (ARHGAP36, FAM171A1, GPCPD1, MT1X, ZNF415, and RXRG) were identified by LASSO analysis. Finally, the validation AUC values indicated that the six diagnostic biomarkers had high diagnostic accuracy for sarcopenia.

**Conclusion:**

We identified six diagnostic biomarkers with high diagnostic performance, providing new insights into the incidence and progression of sarcopenia in future research.

## 1. Introduction

The increasing growth of the aging population has caused much discussion about the impact of aging on public health. Sarcopenia is a common chronic disease with a significant decrease in skeletal muscle mass due to an imbalance between protein synthesis and protein degradation, resulting in a tremendous public health burden. Sarcopenia was defined by Rosenberg in 1989 as a loss of muscle mass, derived from the Greek words Sarx (meat) and Penia (loss), after comparing lean mass in the thighs of an older and younger woman [1]. Although sarcopenia is not a direct cause of death, it can have a pronounced impact on the quality of life in older adults. Loss of skeletal muscle function is an inevitable event in the normal aging process, increasing the risk of adverse outcomes, such as falls, fractures, physical disability, and death [2]. A recent survey found that the prevalence of sarcopenia was 11% and 9%, respectively, among men and women living in the community, but as high as 51% and 31% in nursing homes [3]. Although the incidence of sarcopenia is high, researchers have begun to realize its importance in recent years. In 2016, sarcopenia was listed as a unique disease in the International Classification of Diseases 10, with the code M62.84, according to the 10th edition of the International Statistical Classification of Diseases and Related Health Problems [4].

The pathogenesis of sarcopenia has not been completely clarified, and the mechanism is relatively complex. The balance between skeletal muscle protein synthesis and breakdown can be influenced by age, gender, exercise, and nutritional status [5]. In addition, a variety of factors are known to be involved in the pathogenesis of sarcopenia, such as systemic inflammation, excess glucocorticoids, abnormally increased mitochondria, motor neuron loss associated with accelerated aging, excessive apoptosis, and decreased satellite cell activity [6]. However, the molecular mechanisms of these factors in the development and progression of sarcopenia remain unclear. Although sarcopenia was identified as a new disease state in 2016, the current lack of a functional “gold standard” for sarcopenia diagnosis was not conducive to early screening and prevention of the disease problems in the community. Currently, various methods, including dual-energy X-ray absorptiometry (DEXA), bioelectrical impedance analysis (BIA), magnetic resonance imaging (MRI), and computed tomography (CT), are used to assess skeletal muscle mass. Unfortunately, there is no consensus on the optimal measurement of skeletal muscle mass, especially clinically. Besides, the Foundation for the National Institutes of Health (FNIH) Sarcopenia Project proposed new criteria for defining sarcopenia in terms of muscle mass, strength, and performance [7].

An in-depth study of molecular pathology can better understand the skeletal muscle aging process and contribute to the early diagnosis and prevention of sarcopenia. Recently, microarray technology has been widely used for robust genetic engineering to identify potential novel biomarkers and their roles in various diseases, leading to the further development of potential therapeutics. Zhang and Horvath codeveloped the technique of weighted gene coexpression network analysis (WGCNA) in 2005 [8]. WGCNA can be used not only to construct coexpression networks based on coding RNA data to associate gene modules with clinical features for identifying critical genes but also to construct noncoding RNA networks. By analyzing tens of thousands of genes, WGCNA can cluster genes into coexpression modules according to correlations among their expression pattern and identify gene modules related to the clinical characteristics of samples. Therefore, we utilized differential expression analysis and WGCNA to find key genes associated with sarcopenia, which would help to elucidate the molecular mechanism of aging-induced sarcopenia. Moreover, the diagnostic biomarkers in the key genes were selected using the least absolute shrinkage and selection operator (LASSO). LASSO, applied to pick out predictor candidates, is a valuable approach for reducing and selecting high-dimensional data [9]. Our research is aimed at identifying the hub genes and functional enrichment pathways responsible for the development and progression of sarcopenia and determining effective biomarkers and therapeutic targets for sarcopenia.

## 2. Materials and Methods

### 2.1. Research Design

In order to obtain a larger sample size, three microarray expression datasets were merged and batch corrected, and differentially expressed genes (DEGs) between the normal group and sarcopenia group in the merged dataset were identified. Meanwhile, we performed WGCNA on the merged dataset to obtain a coexpression gene module associated with clinical characteristics. The intersection between the DEGs and the genes in the coexpression gene module was defined as common genes (CGs). Then, we performed functional enrichment analysis and protein-protein interaction (PPI) network to explore the role of CGs in the pathogenesis of sarcopenia. Besides, 15 hub genes were identified using LASSO logistic regression, and their diagnostic performance was assessed by receiver operating characteristic (ROC) analysis. Subsequently, a novel diagnostic nomogram model based on the hub genes with the area under the curve (AUC) values exceeding 0.9 was constructed to screen and predict sarcopenia. Finally, ROC analysis was used to further assess and validate the prediction capability of the hub genes and the nomogram model in external-validation datasets.

### 2.2. Data Acquisition and Preprocessing

Firstly, four microarray expression datasets (GSE38718, GSE8479, GSE9103, and GSE28422) and one RNA sequencing dataset (GSE111016) from the National Center for Biotechnology Information Gene Expression Omnibus database (NCBI-GEO; https://www.ncbi.nlm.nih.gov/geo/) were obtained with the keywords “sarcopenia”. GSE38718 consisted of eight sarcopenia samples and fourteen normal samples; GSE8479 consisted of 51 skeletal muscle tissue samples, including 25 sarcopenic samples and 26 normal samples; GSE9103 consisted of 20 skeletal muscle tissue samples of ten patients with sarcopenia and ten normal samples. A total of 12 sarcopenic samples and 15 normal samples were included in GSE28422; GSE111016 consisted of 20 sarcopenia samples and 20 normal samples (see Table 1 for details). Secondly, three of the GEO datasets (GSE38718, GSE8479, and GSE9103) were merged into one gene expression matrix file as the training dataset, which was batch normalized by using the “sva” package of the R software [10]. Finally, a normalized gene expression matrix file was obtained for differential gene expression analysis and weighted gene correlation network analysis. Additionally, GSE28422 and GSE111016 served as the validation datasets to test the diagnostic performance of hub genes and the nomogram model.

### 2.3. DEG Analysis

The merged dataset consisted of 50 normal samples (24 males and 26 females) and 43 senile sarcopenia samples (21 males and 22 females). Besides, all muscle biopsy samples were obtained from the vastus lateralis muscle. The “limma” package of the R software was used to analyze DEGs in the merged dataset [11]. In this study, genes that met double filtering criteria were considered DEGs: absolute log2 − fold change > 0.5 and Benjamini-Hochberg false discovery rate (FDR), adjusted *P* value ≤ 0.05. The DEGs were visualized using the R packages “ggplot2” and “pheatmap” [12, 13] to generate volcano distribution maps and heatmaps, respectively.

### 2.4. WGCNA Construction and Module Identification

WGCNA builds gene coexpression networks by correlating gene expression levels with clinical features and is widely used to study potential interactions between genes. The study applied the R package “WGCNA” [8] to construct a coexpression network between sarcopenia and normal samples. First, genes exceeding 25% intersample variation in the merged dataset were imported into the WGCNA package. We removed outlier samples from the training dataset to obtain accurate and reliable results. Then, an adjacency value was calculated by using the pick-Soft-Threshold function, which preserved soft-threshold power based on coexpression similarity. Subsequently, adjacency values were converted to topological overlap matrices (TOM), and the corresponding dissimilarity (1-TOM) was figured out. Third, the topological overlap matrix was hierarchically clustered using the average algorithm, and the gene modules were detected using dynamic tree cutting. Fourth, we limited the minimum number of genes per module to 50 and merged strongly correlated modules with a threshold of 0.4 to obtain correlated modules. Next, the correlations between genes and clinical features in each module were determined by calculating gene significance and module membership (MM). In the end, the distinct gene network was visualized. Meanwhile, the intersection of the DEGs and the genes from the module most significantly correlated with clinical features was defined as CGs.

### 2.5. Functional Enrichment Analysis

To further reveal the characteristic biological properties of CGs, we used the “clusterProfiler” package in R software [14] and Metascape (http://metascape.org) to perform functional enrichment analysis, including gene ontology (GO) analysis and Kyoto Encyclopedia of Genes and Genomes (KEGG) pathway analysis. GO terms were grouped into major categories, including molecular function (MF), biological process (BP), and cellular component (CC). Terms with the corrected threshold of *P* < 0.05 were considered significantly enriched by CGs. Multiseries chord graphs for the top ten GO terms of CGs were created using the “ggplot2” and “GOplot” packages in R [15]. Bubble and bar charts were generated using the “ggplot2” and “clusterProfiler” packages of R to visualize the KEGG enrichment analysis of CGs.

### 2.6. LASSO Regression Analysis and Assessment of the ROC Curve

As a machine learning technique, LASSO regression analysis was used to identify a variable by detecting the optimal *λ* value with the lowest classification error. LASSO analysis was performed to screen the CGs using the R package “glmnet” [16] with a response type of binomial and an alpha of 1. Then, the hub genes of sarcopenia were identified using LASSO regression analysis, and 10-fold cross-validation was applied to choose the optimal value of penalty parameter *λ*. Moreover, ROC curves were plotted for hub genes of sarcopenia by using the “pROC” package of R [17]. The diagnostic power of the hub genes was evaluated by the AUC of the ROC curve. AUC values lower than 0.7 were defined as the discriminant value of the difference; AUC values of 0.7 to 0.8 were the lower limit of accuracy; AUC values of 0.8 to 0.9 indicated excellent discrimination. The hub genes with the AUC values exceeding 0.9 were considered as diagnostic biomarkers of sarcopenia due of their outstanding discrimination. The optimal cut-off point for this ratio was chosen based on the Youden index and the confidence interval estimated at its 95% confidence limit (CI).

### 2.7. Verification of Diagnostic Biomarkers

To judge the accuracy of the diagnostic biomarkers, we used an external dataset (GSE28422) as a testing dataset to validate the diagnostic and predictive performance. The ROC curve of GSE28422 was generated using the “pROC” package of R, and the AUC and 95% CI were used to validate the model efficiency. Furthermore, the Wilcoxon rank-sum test was used to compare the differences in the gene expression level of diagnostic biomarkers between sarcopenia and normal muscle samples. Ultimately, a violin plot was generated for visualization by the “vioplot” package in R.

### 2.8. Evaluation and Verification of the Nomogram Model

Based on the selected diagnostic biomarkers of sarcopenia, a novel diagnostic nomogram model was constructed using the R package “rms” to predict the prevalence of sarcopenia patients. ROC curve of the model on the training dataset and the RNA sequencing dataset (GSE111016) were drawn by using the “pROC” package of R to calculate the AUC for judging the accuracy of the model.

### 2.9. Statistical Analysis

All statistical analyses were applied using R software (R version 4.1.3). The Wilcoxon rank-sum test compared the differences between sarcopenia and the normal group. Corresponding 95% CIs were reckoned with confidence interval estimation, and *P* < 0.05 was statistically significant.

## 3. Results

### 3.1. Screening of DEGs

Using the “limma” package of the R software, 107 DEGs were screened in a combined dataset of 43 elderly patients with sarcopenia and 50 normal controls. DEGs included 46 low-expressed genes and 61 highly expressed genes, including SLPI and MYH8 with log FC > 1. The results of DEGs were visualized in the volcano map and heatmap (Figure 1). The top five most significantly upregulated genes were SLPI, MYH8, ADIRF, MT1X, and LRP1B, while the top five most significantly downregulated genes were RXRG, GADD45G, SLC38A1, SCN4B, and KLHL34. The abundance of DEGs have been provided in the supplementary material (Supplementary Table 1).

### 3.2. Identification of Sarcopenia-Related Modules and Genes

First, the genes were sorted based on the variance from large to minor, and the top 25% of genes were selected for subsequent analysis. A total of 3859 genes were obtained in the first step. Second, we clustered the samples using the flashClust module, and one outlier sample was discovered from our analysis by setting the threshold value to 45 (Figure 2(a)). Third, the power parameter values ranging from 1 to 20 were filtered out using the pick-Soft-Threshold function. The soft-threshold power value of 4 was determined according to the scale-free topology criterion for network construction (Figure 2(b)). By setting the threshold to 0.4 to merge similar modules in the hierarchical cluster tree, 11 gene modules (marked with different colors) were finally identified (Figure 3(a)).

Coexpression network analysis revealed that the module eigengenes in the turquoise module (*r* = −0.81, *P* = 2*e* − 22) exhibited the highest negative correlation with sarcopenia (Figure 3(b)). Therefore, the turquoise module was defined as the sarcopenia-related module, and 788 genes in this module were defined as sarcopenia-related genes (Figure 3(c)). After overlapping sarcopenia-related genes and DEGs, 72 genes were selected as CGs of sarcopenia for further analysis.

### 3.3. Functional Enrichment Analysis and PPI Network of CGs

GO enrichment analysis of CGs yielded 269 enriched annotations, including 260 BPs and 9 CCs. The details of 269 enriched annotations are provided in supplementary material (Supplementary Table 2). The top five most significant GO terms of BP and CC were shown in the circle and chord plots (Figures 4(a) and 4(b)). BP analysis revealed that CGs were mainly enriched in the animal organ regeneration, the detoxification of copper ions and inorganic compounds, and stress response to metal ions. Among the CC category, CGs are mainly involved in mitochondria's inner and part membrane, the protein complex in mitochondria and inner mitochondrial membrane, and myosin filament (see Table 2 for details). We also performed the KEGG pathway enrichment analysis on CGs. The results showed that CGs were mainly enriched in the mineral absorption, glucagon signaling pathway, FoxO signaling pathway, insulin signaling pathway, AMPK signaling pathway, and estrogen signaling pathway. The top 11 most significant KEGG pathways involved by the CGs are shown in Figures 4(c) and 4(d).

### 3.4. Evaluation of Diagnostic Value of Hub Genes by LASSO Analysis

The expression profiles of 72 CGs were extracted for building the LASSO model. As shown in Figure 5(a), the optimal *λ* (*λ* = 15), which produced the minimum classification errors, was determined in the LASSO model. Based on the *λ* value of 15, the LASSO coefficient spectrum of CGs was screened out (Figure 5(b)). Subsequently, 15 hub genes with nonzero coefficients were identified, including FAM171A1, ZNF415, MT1X, C6orf136, GPCPD1, RXRG, ARHGAP36, SCN4B, HOXB2, ATP1B4, NEDD1, TGFBR3, MT2A, KLF5, and TXNIP. Moreover, the ROC curves and AUC values were generated to evaluate the diagnostic performance of 15 hub genes. Finally, six hub genes with AUC exceeding 0.9, including GPCPD1, MT1X, ARHGAP36, FAM171A1, ZNF415, and RXRG, were defined as diagnostic biomarkers of sarcopenia (Figure 6). The specific information on the diagnostic efficacy of 15 hub genes is shown in Table 3.

### 3.5. Validation of the Diagnostic Biomarkers

An external dataset (GSE28422) was used to validate the six diagnostic biomarkers to judge whether the biomarkers could distinguish sarcopenia samples from normal samples. As shown in Figure 7, we found the AUC values of GPCPD1, MT1X, ARHGAP36, FAM171A1, ZNF415, and RXRG on the validation dataset were 0.928, 0.75, 0.978, 0.961, 0.811, and 0.906, indicating that the six biomarkers had high diagnostic accuracy for sarcopenia. Besides, to further validate the gene expression levels of the six diagnostic biomarkers, we performed the differential expression analysis in the training and validation datasets, respectively (Figure 8). Compared to normal samples, the expression levels of both MT1X and ARHGAP36 were upregulated in sarcopenia samples, while GPCPD1, FAM171A1, ZNF415, and RXRG showed lower expression in sarcopenia samples. Consistent with our predictions, the gene expression differences of the six diagnostic biomarkers between sarcopenia and normal samples were statistically significant, both in the training and validation datasets.

### 3.6. Construction and Verification of the Diagnostic Nomogram Model

Based on the six diagnostic biomarkers, we established a nomogram model to predict the onset of sarcopenia (Figure 9). The nomogram model predicted an AUC of 1 on the training dataset (Figure 10(a)) and an AUC of 0.9 on the test dataset (GSE111016) (Figure 10(b)), indicating that the nomogram model had high classification performance. The results showed that we successfully constructed a diagnostic model for sarcopenia from the differential gene expression of the six diagnostic biomarkers.

## 4. Discussion

Loss of muscle mass and function in the elderly is a growing public health problem with increasing longevity. Therefore, early prediction and diagnosis of sarcopenia increase the possibility of intervention. Unluckily, there are no internationally accepted criteria for diagnosing sarcopenia. Hence, searching for potential diagnostic biomarkers is crucial for the early diagnosis and screening of sarcopenia in the community population. Instead of focusing on the phenotypic diagnosis, we used WGCNA and LASSO analysis to further identify novel diagnostic biomarkers of sarcopenia that showed significant advantages in gene selection and classification. To our knowledge, our research is the first reported in the literature combining WGNCA and LASSO analysis to identify potential diagnostic biomarkers for sarcopenia.

In recent years, the availability of gene expression data in public databases has created new diagnostic and predictive options for sarcopenia. Thus, we performed a comprehensive analysis of sarcopenia using various GEO datasets and applied bioinformatics to obtain potential diagnostic biomarkers. Firstly, 107 DEGs were identified in the merged dataset through differential expression analysis. Among them, the expression levels of SLPI and MYH8 in the sarcopenia group were significantly higher than those in the normal group (log2 FC > 1). Secretory leukocyte peptidase inhibitor (SLPI), encoded by the SLPI gene, acts as an inhibitor of nuclear factor-*κ*B (NF-*κ*B), binding to IL-8 and tumor necrosis factor-*α* (TNF-*α*) sites on the promoter [18]. In recent years, the notion that inflammation is involved in the pathogenesis of age-related sarcopenia has gained increasing acceptance in the scientific community. The primary effect of inflammation on sarcopenia is achieved by activating the NF-*κ*B pathway. As the most potent activator of the NF-*κ*B pathway, TNF-*α* promotes positive feedback by activating NF-*κ*B, which in turn induces TNF*α* and leads to NF-*κ*B-mediated muscle atrophy [19]. Therefore, the high gene expression of SLPI in the sarcopenia group might indicate the importance of inflammation in the pathogenesis of sarcopenia. Increased expression of myosin heavy chain 8 (MYH8) is a hallmark of muscle recovery [20]. MYH8, a component of myosin, is mainly expressed in neonatal skeletal muscle [21]. In certain pathological conditions, progenitor cells can proliferate and differentiate into muscle cells during skeletal muscle regeneration but do not develop during fiber maturation [22].

In addition to the difference analysis, we also performed WGCNA in the merged dataset to select the gene module that closely corresponded to the occurrence of sarcopenia. Furthermore, 72 CGs were identified by overlapping the genes obtained by the WGCNA and differential expression analysis. BP analysis showed that these CGs were mainly involved in the stress response and detoxification of metal ions (especially copper ions). These results led us to hypothesize that copper ions may accumulate in the skeletal muscle cells of sarcopenia patients. Tsvetkov et al. [23] have found that copper ions are directly bound to fatty acid acylated components in the tricarboxylic acid cycle, resulting in the abnormal aggregation of fatty acid acylated proteins and loss of iron-sulfur cluster proteins. Thence, copper-induced cell death may be an essential mechanism for developing sarcopenia and requires further investigation. On the other hand, CC analysis revealed that CGs were mainly involved in mitochondrial structure and the composition of the mitochondrial-associated protein complex. It is well-known that mitochondria, as an organelle, have various biological functions in cells. Given that mitochondria are the most important organelles in the regulation of energy generation and that skeletal muscle is the main energy-generating organ of the body, mitochondria are the key organelles for oxidative metabolism in the skeletal muscle [24]. Therefore, mitochondrial dysfunction is believed to play a central role in the underlying mechanism behind sarcopenia [25]. Based on the results of CC analysis in this study, we believed that mitochondrial structure disruption and impairment of mitochondrial protein complex synthesis, inducing mitochondrial dysfunction, might exist in the skeletal muscle of sarcopenia patients.

Through the KEGG pathway enrichment analysis, these CGs were mainly involved in AMPK and FoxO signaling pathways closely associated with the pathogenesis of sarcopenia. AMP-activated protein kinase (AMPK) is an essential regulator of mitochondrial skeletal muscle function and oxidative stress and is involved in regulating multiple cellular functions [26]. Activation of AMPK modulates signaling pathways related to energy metabolism, promotes mitochondrial biosynthesis, and improves skeletal muscle dysfunction during aging [27]. Therefore, activating the AMPK pathway may maintain skeletal muscle mass by affecting mitochondrial biogenesis and mitochondrial structural protein synthesis. Forkhead box transcription factors (FoxO) are widely distributed in several eukaryotes, including FoxO1 and FoxO3a in the skeletal muscle [28]. FoxO1 and FoxO3a proteins transcriptionally upregulate the expression of the muscle-enriched E3 ubiquitin ligase associated with sarcopenia, including muscle RING finger 1 and muscle atrophy F-box [29].

In this research, 15 CGs were identified as hub genes for sarcopenia via LASSO analysis (see Table 3). Moreover, six hub genes with AUC exceeding 0.9, including ARHGAP36, FAM171A1, GPCPD1, MT1X, ZNF415, and RXRG, were confirmed as diagnostic biomarkers for sarcopenia. ARHGAP36 (Rho GTPase Activating Protein 36) encodes a protein belonging to the Rho-GAP family and acts as a positive regulator of sonic hedgehog (SHH) signaling by activating Gli protein [30]. As a critical transcriptional regulator of SHH signaling, Gli protein directly controls the expression of myogenic regulatory factor 5 (Myf5) in muscle progenitors, which promotes the differentiation of mesoderm cells into distinct myogenic lineages [31]. We speculated that ARHGAP36 might be involved in skeletal muscle differentiation by mediating SHH signaling in skeletal muscle progenitor cells. FAM171A1 (family sequence similarity 171, member protein A1) is an 890 amino acid glycoprotein expressed in placental trophoblasts, skeletal muscle, kidneys, and pancreas [32]. Since FAM171A1 was discovered recently, there is little existing information about FAM171A1 in the literature. The research conducted by Rasila et al. [32] was the first to report the functional properties of FAM171A1 in regulating tumor cell morphology and aggressive growth potential of tumor cells by modulating actin cytoskeleton dynamics. Further investigations are needed to reveal other functional characterizations of FAM171A1, and the role of FAM171A1 in the pathogenesis of sarcopenia would be an important future research direction.

GPCPD1 encodes glycerophosphodiester phosphodiesterase 5 (GDE5), a key enzyme in choline phospholipid metabolism, highly expressed in fast skeletal muscle fibers [33]. Hashimoto et al. [34] found that transgenic mice overexpressing GDE5dC471, a truncated mutant of GDE5 without phosphodiesterase activity, displayed less skeletal muscle mass than control mice. However, Okazaki et al. pointed out that GDE5 inhibited skeletal muscle differentiation [35]. In the present study, we found that the gene expression of GPCPD1 in muscle samples from patients with sarcopenia was significantly lower than that in normal samples (Figure 8), indicating that GPCPD1 might have the effect of inhibiting muscle atrophy. The mechanism by which GPCPD1 regulates skeletal muscle development requires further investigation. MT1X encodes metallothionein-1X, a functional (sub)isoform of MT1 [36]. Metallothionein proteins are small, cysteine-rich metal-binding proteins that play important roles in maintaining cellular homeostasis and detoxifying transition metals [37]. Overexpression of MX1X in aged skeletal muscle suggests that the presence of metal ion overload deposits may be involved in the development of sarcopenia. Zinc finger protein 415 encoded by ZNF415, a novel protein with p53 inhibitory activity, was first discovered in the human fetal cDNA library in 2006 [38]. As a central regulator of the cell cycle and apoptosis, p53 is considered to regulate skeletal muscle homeostasis and atrophy during aging [39]. Therefore, ZNF415 may reduce myocyte apoptosis by inhibiting the P53 pathway, thereby delaying the occurrence and development of muscle atrophy.

Despite many revolutionary discoveries, there are still some limitations. First, all muscle samples were sourced from the GEO database. Although we performed external validation to support the diagnostic efficacy of six identified diagnostic biomarkers, no proprietary experimental data were available for validation. Second, the merged dataset was a combination of three small sample size datasets. Although the batch effect has been removed, it is still not the most suitable dataset. Nevertheless, our discovery of proteins encoded by these crucial genes may serve as characteristic biomarkers and provide specific insights for future diagnosis and screening of sarcopenia.

## 5. Conclusion

In this research, six genetic biomarkers closely associated with sarcopenia, including ARHGAP36, FAM171A1, GPCPD1, MT1X, ZNF415, and RXRG, were identified by WGNCA and LASSO analysis, which were used to future diagnose and screen for sarcopenia.

## Figures and Tables

**Figure 1:** (a) Volcano plot of DEGs. The red dots in the upper right part represent upregulated DEGs. The blue dots in the upper left part represent downregulated DEGs. The middle black dots represent the remaining stable genes. (b) Heatmap of the top 60 DEGs. The colors from red to green in the figure represent the expression of DEGs from high to low.

**Figure 2:** (a) Sample cluster analysis was applied to detect outliers. The threshold value was set to 45, removing 1 outlier sample. (b) Analysis of network topology was used to acquire the scale-free fit index.

**Figure 3:** Weighted gene coexpression network analysis. (a) Different modules in the gene coexpression network represented by different colors under the gene tree. (b) Heatmap of the association between modules and sarcopenia. *P* values and correlation coefficients are represented by numbers inside and outside parentheses, respectively. (c) Correlation chart between MM and GS of the clustered genes in the turquoise module.

**Figure 4:** Functional and pathway enrichment analyses of common genes (CGs) at the intersection. (a) Circle plot showing GO terms. The circle inside represented *Z*-score. The dots in the middle represented CGs: blue represents downregulated CGs, and red represents upregulated CGs. The outer circle represented different GO terms. (b) Chord plot showing GO terms. CGs were indicated on the left. The different colored bands on the right represent different GO terms. Connecting lines indicate that the gene is enriched in the GO terms. (c) Bubble graph of KEGG pathway enrichment results. The size of the bubble represents the number of DEGs enriched in the KEGG pathways. (d) Bar graph of KEGG pathway enrichment results. The *X* axis represents the *q* value (-log10), and the *Y* axis represents the KEGG pathways.

**Figure 5:** The potential hub genes of sarcopenia were identified by the LASSO regression model. (a) Selection of the best parameter of nonzero coefficients in the LASSO model; (b) LASSO-based coefficient selection of 15 hub genes by optimal.

**Figure 6:** ROC curves of diagnostic biomarkers with AUC exceeding 0.9 on the training dataset. (a–f) ROC curves for GPCPD1, MT1X, ARHGAP36, FAM171A1, ZNF415, and RXRG, respectively.

**Figure 7:** ROC curves of diagnostic biomarkers on the validation dataset (GSE28422). (a–f) ROC curves for GPCPD1, MT1X, ARHGAP36, FAM171A1, ZNF415, and RXRG, respectively.

**Figure 8:** Violin plots showed gene expression differences of the six diagnostic biomarkers between normal and sarcopenia groups in the training dataset (a, b) and validation dataset (c, d). The red box reflected the sarcopenia group, and the green box reflected the normal group. ^∗^*P* < 0.05, ^∗∗^*P* < 0.01, and ^∗∗∗^*P* < 0.001.

**Figure 9:** The nomogram model of sarcopenia.

**Figure 10:** ROC curve of the nomogram diagnostic model of sarcopenia on the combined dataset (a) and the RNA-seq dataset (b).

**Table 1:** Source of GEO datasets.

GEO datasets	Platform	Sarcopenia samples	Normal samples
Train group			
GSE38718	GPL570	8	14
GSE8479	GPL2700	25	26
GSE9103	GPL570	10	10
Test group			
GSE28422	GPL570	12	15
GSE111016	GPL16791	20	20

**Table 2:** The top five of each biological process and cellular component by fold enrichment and significance from GO-term analysis of CGs.

ID	GO terms	Gene symbol involved in the pathway	*P*.adjust
Biological process			
GO:0031100	Animal organ regeneration	CEBPB/TGFBR3/NNMT/PKM/CDKN1A	4.33*E*-06
GO:0010273	Detoxification of copper ion	MT1X/MT1H/MT2A	1.54*E*-05
GO:1990169	Stress response to copper ion	MT1X/MT1H/MT2A	1.54*E*-05
GO:0061687	Detoxification of inorganic compound	MT1X/MT1H/MT2A	2.29*E*-05
GO:0097501	Stress response to metal ion	MT1X/MT1H/MT2A	2.29*E*-05
Cellular component			
GO:0044455	Mitochondrial membrane part	PPIF/APOO/TOMM40L/CISD1/IMMT/NDUFA3/COX7A2	1.13*E*-05
GO:0005743	Mitochondrial inner membrane	PPIF/APOO/CKMT2/COQ10A/IMMT/NDUFA3/COX7A2	0.001005
GO:0098800	Inner mitochondrial membrane protein complex	PPIF/APOO/IMMT/NDUFA3	0.001091
GO:0098798	Mitochondrial protein complex	PPIF/APOO/TOMM40L/IMMT/NDUFA3	0.001841
GO:0032982	Myosin filament	MYH8/MYOM2	0.002441

**Table 3:** Evaluation of hub gene diagnostic capabilities.

Gene symbol	Sensitivity (%)	Specificity (%)	AUC	95% CI	Youden index
FAM171A1	0.837	0.94	0.929	0.874-0.985	0.777
ZNF415	1	0.66	0.925	0.875-0.974	0.66
MT1X	0.93	0.84	0.932	0.880-0.983	0.77
C6orf136	0.767	0.82	0.83	0.743-0.917	0.587
GPCPD1	0.86	0.84	0.912	0.856-0.968	0.7
RXRG	0.907	0.76	0.92	0.868-0.972	0.667
ARHGAP36	0.791	0.96	0.91	0.851-0.969	0.751
SCN4B	0.814	0.8	0.865	0.793-0.938	0.614
HOXB2	0.837	0.9	0.888	0.812-0.964	0.737
ATP1B4	0.86	0.76	0.87	0.796-0.943	0.62
NEDD1	0.721	0.86	0.833	0.750-0.917	0.581
TGFBR3	0.814	0.72	0.833	0.749-0.918	0.534
MT2A	0.814	0.68	0.799	0.711-0.888	0.494
KLF5	0.791	0.8	0.847	0.765-0.928	0.591
TXNIP	0.674	0.68	0.712	0.608-0.816	0.354

## Data Availability

Data supporting the findings of this research are available from the corresponding author upon request.

## Supplementary Materials

Supplementary Materials Table S1: the details of 107 DEGs. Table S2: the details of 269 GO enrichment analysis of CGs.
